This article has been retracted.

# The Role of microRNAs in the Tumorigenesis of Ovarian Cancer

**DOI:** 10.3389/fonc.2013.00153

**Published:** 2013-06-13

**Authors:** Gianpiero Di Leva, Carlo M. Croce

**Affiliations:** ^1^Department of Molecular Virology, Immunology, and Medical Genetics, Comprehensive Cancer Center, The Ohio State University Columbus, OH, USA

**Keywords:** microRNA, ovarian cancer, noncoding RNA, miRNA profiling, miRNA profiles

## Abstract

Epithelial ovarian cancer (EOC) is a complex disease, with multiple histological subtypes recognized. There have been major advances in the understanding of the cellular and molecular biology of this human malignancy, however the survival rate of women with EOC has changed little since platinum-based-treatment was introduced more than 30 years ago. Since 2006, an increasing number of studies have indicated an essential role for microRNAs (miRNAs) in ovarian-cancer tumorigenesis. Several miRNA profiling studies have shown that they associate with different aspects of ovarian cancer (tumor subtype, stage, histological grade, prognosis, and therapy resistance) and pointed to a critical role for miRNAs in the pathogenesis and progression of EOC. In this review, we discuss the current data concerning the accumulating evidence of the modulated expression of miRNAs in EOC, their role in diagnosis, prognosis, and prediction of response to therapy. Given the heterogeneity of this disease, it is likely that increases in long-term survival might be also achieved by translating the recent insights of miRNAs involvement in EOC into novel targeted therapies that will have a major impact on the management of ovarian cancer.

## Introduction

Among United States women, ovarian cancer is the sixth most common cancer and the second most common gynecologic cancer (after endometrial cancer) (Parkin et al., 2002). Ovarian-cancer occurs in 1 of 2500 postmenopausal women in the United States and accounts for 5–6% of all cancer-related deaths (Jemal et al., 2008). The 5-year survival rate of ovarian-cancer ranges from 30 to 90%, depending on the spread of disease at diagnosis. When ovarian cancer is diagnosed at early stages, the survival rate is close to 90%; unfortunately, the vast majority of patients is identified when they have late-stage disease (Goff et al., 2000). This is primarily because ovarian cancer has few early or specific symptoms shared with many more common gastrointestinal, genitourinary, and gynecological conditions and have not yet proved useful for early diagnosis. Patients diagnosed with advanced disease are managed with surgical cytoreduction and chemotherapy, but many experience resistance to chemotherapy and relapse, yielding an overall 5-year survival rate of 10–30%. At the cellular and molecular levels, ovarian cancers are remarkably heterogeneous (Boxes 1 and 2). The normal ovary is a complex tissue with several distinct components. Although ovarian cancers can develop from germ cells or granulosa-theca cells, more than 90% of ovarian cancers have an epithelial histology and are thought to arise from cells that cover the ovarian surface or that line subsurface inclusion cysts (Feeley and Wells, 2001). One of the major disappointments in the field of ovarian-cancer research is the failure of currently established therapies to induce a cure at diagnosis, even in chemosensitive tumors. Efforts have been made to cure ovarian cancer over the past decade using different classes of chemotherapeutic agents in various combinations, dosages, and schedules to overcome chemoresistance following front-line paclitaxel–platinum treatment. Our improved understanding of the underlying biology of ovarian tumor etiology and chemoresistance has led to the development of molecular targeted therapies. Many small-molecule inhibitors and monoclonal antibodies that target multiple crucial cancer characteristics, including cell growth and survival, angiogenesis, and metastases are now entering clinical trials (Figure 1). However, new efforts are needed to identify new and better markers/therapeutics to aid the diagnostic and curative process of ovarian cancer.

Box 1 **Ovarian-cancer subtypes.**

Despite the controversy surrounding the histogenesis of ovarian cancers, it is widely believed today that most OECs (90%) arise from the ovarian surface epithelium. OECs are now classified in several histologic subtypes with distinctive risk factors, genetic abnormalities, and oncologic pathways that partly determine biologic behavior, response to chemotherapy, and prognosis. OECs develop from simple flattened epithelial cells into four different main histotypes that resemble the well-differentiated cells of the fallopian tube (serous, the most common with 7 out of every 10 epithelial ovarian cancers), endometrium (endometrioid, 1 in 20 epithelial ovarian cancers), endocervix (mucinous, 1 in 10 epithelial ovarian cancers), and cells that form nests within the vagina (clear cells, the least common subtype of epithelial ovarian cancer with just 3 in 100 cases). A significant proportion of endometrioid carcinomas and clear-cell carcinomas is associated with preexisting endometriosis. Serous carcinoma can be classify in high-grade (HGSC) and low-grade tumors (LGSC). Most HGSCs are biologically aggressive neoplasms, and they often manifest at an advanced stage, with up to 85% of patients with ovarian serous carcinoma presenting with widespread peritoneal metastases. Up to 80% of HGSCs show initial response to platinum-based chemotherapy, but about 70% may demonstrate recurrence. LGSC behaves like a slow-growing indolent neoplasm (presumably due to lack of p53 mutations) and has a better prognosis. Unlike HGSCs, recurrent LGSCs have high extreme drug resistance to paclitaxel, carboplatin, and cisplatin (33–69% of cases), but low drug resistance to etoposide and doxorubicin. Endometrioid carcinomas are platinum-sensitive tumors and, owing to low-grade early-stage disease and better chemotherapy sensitivity, are associated with the most favorable prognosis among all subtypes of EOCs. Mucinous neoplasms account for 10–15% of all ovarian tumors and up to 80% of mucinous neoplasms are benign cystadenomas. Clear-cell carcinomas are biologically aggressive neoplasms despite their being diagnosed at early stages. In this case, recurrence following surgery is common. Clear-cells and mucinous cancers generally do not respond as well as serous and endometrioid cancers to platinum- and taxane-based chemotherapy.

Box 2 **Ovarian-cancer genomic alteration.**

At molecular levels, the gene expression profiles of the different ovarian-cancer histotypes correlate with their morphological counterparts in normal tissues. HGSC is frequently characterized by mutations or loss of heterozygosity of p53 and genetic-epigenetic silencing of BRCA genes (∼80% of cases). Instead, LGSCs are characterized by frequent mutations of K-ras, BRAF, and erb-B2 (HER-2) genes. In endometrioid carcinomas CTNNB1 mutations (38–50% of cases), PTEN mutations (20%), and microsatellite instability (up to 19%) are commonly seen. In mucinous carcinomas, K-ras mutations are common and constitute an early event in tumorigenesis. Moreover, HER-2 gene amplification is seen in 15–20% of tumors. Clear-cell carcinomas are the most common histologic subtype characterized by the highest frequency of PI3KCA mutations: 33% of these carcinomas demonstrate activating mutations of PI3KCA. Mutations involving the PIK3CA gene lead to activation of the PI3K/AKT pathway, resulting in improved cell survival and invasion. The different histotypes of EOCs have also been correlated with the abnormal re-expression of homeobox genes (HOX) that are normally expressed during the formation of gynecological organs. HOXA9 is highly expressed in serous, HOX 10 in endometrioid, and HOXA11 in mucinous ovarian cancer. The vast majority of OECs (90%) are sporadic, with the remainder being inherited as part of hereditary ovarian-cancer syndromes. Germline mutations of BRCA1 and BRCA2 tumor-suppressor genes are responsible for most hereditary ovarian cancers (90–95%). The lifetime risk of developing ovarian cancer is about 20–50% in patients carrying BRCA mutations.

**Figure 1:** **Signaling pathways and new therapeutic targets for ovarian cancer**. Despite many efforts in these last few years, clinical responses to curative chemotherapy in ovarian cancer remain very low and have merely led to improvements in the survival of patients. Therefore, new different drugs and combination treatments have been identified and are now entering clinical trials to test new therapeutic possibilities. In the figure, we depicted in blue some of the most important new or promising clinical targets in ovarian cancers. Many other different therapeutic approaches have also been taken and here not depicted, such as new cytotoxic agents (trabectedin, patupilone, canfosfamide), anti-folate transporter 1 inhibitor (farletuzumab), PARP inhibitor (olaparib).

MicroRNAs (miRNAs) are single-stranded RNAs (ssRNAs) ∼19–25 nt in length that negatively regulate gene expression by translation inhibition or messenger RNA (mRNA) degradation, through base-pairing to partially complementary sites on the target mRNAs, usually in the 3′ untranslated region (UTR) (Garofalo and Croce, 2011; Mendell and Olson, 2012). Bioinformatic analyses predict the existence of ∼1000 miRNAs in the human genome capable to regulate up to 60% of all human transcriptome. Due to their highly abundance, conservation and tissue specific expression miRNAs play key roles in almost all biological processes, including gene regulation, cell developmental control, and the development of various diseases, such as cancer. Dysregulation of miRNA expression appears to play a fundamental role in the onset, progression and dissemination of cancers, and replacement of down-regulated miRNAs in tumor cells results in a positive therapeutic response (Croce, 2009). Accumulating data have shown that miRNAs are also aberrantly expressed in ovarian cancer and can be associated with tumor subtypes, clinical outcomes, and chemoresistance, indicating that miRNAs may be involved in ovarian tumorigenesis and progression. In the following review, we will discuss recent progresses in understanding the functions of miRNAs in ovarian cancer and their possible use as diagnostic and prognostic markers, and eventually as new targets or tools of a specific therapy.

## MicroRNA in Cancer

Over the last 10 years, we have seen an enormous number of studies concerning the role of miRNAs in cancer (8461 PubMed hits on February 2013). Despite the large variety both in terms of the diseases and the experimental approaches taken, many essential and general principles of miRNA activity in human cancer have been defined. miRNAs activity is firstly related to redundancy: each miRNA exerts its full functional effects by regulating hundreds or thousands of targets (Mendell and Olson, 2012). To complicate the scenario, many miRNAs exist in families with similar seed sequences, and many of them from different families are co-expressed as a large clusters to amplify and maximize their inhibitory activity. Redundancy can also be found at the level of the target mRNAs where different miRNAs may also repress the same target. The second important aspect of miRNA/cancer relationship has been revealed by the application of the high-throughput technologies which have allowed the identification of cancer-specific miRNA fingerprints in all type of human cancer (Calin and Croce, 2006; Croce, 2009). In general, the expression of miRNAs in malignant cells is significantly different from that of normal counterpart cells and facilitate the stratification of cancer and the identification of the tissue of origin for poorly differentiated tumors. Some of the most commonly dysregulated miRNAs in cancer are summarized in Table 1. The third essential aspect of miRNA implication in cancer is represented by the fact that miRNAs can be up- or down-regulated in malignancies and, therefore, respectively referred to as oncogenes or tumor suppressors, sometimes even if there is no evidence for their causative role in tumorigenesis (Esquela-Kerscher and Slack, 2006; Croce, 2009). The more characterized and first identified tumor-suppressor miRNA is represented by the miR-15/16 cluster, deleted in 68% of Chronic Lymphocytic Leukemia (CLL) patients carrying a 13q14.3 translocation (Calin et al., 2002). A mouse model that mimics the minimal deletion region 13q14.3 or that specifically deletes the miR-15a/16-1 cluster exhibited a full spectrum of CLL-associated phenotypes, consistent with the miR-15a/16-1 locus having a tumor-suppressor role in the B-cell lineage (Klein et al., 2010). An example of oncogenic miRNA is miR-155, which is overexpressed in different types of B-cell malignancies, including pediatric Burkitt’s lymphoma, Hodgkin’s lymphoma, aggressive CLL, and diffuse large B-cell lymphoma (DLBCL) (Croce, 2009). Transgenic expression of miR-155 is sufficient to initiate lymphomagenesis in mice (Costinean et al., 2006). Another aspect to be considered is the high context-dependent activity of miRNAs. The same miRNA can act as an oncogene in one type of cells and as a tumor suppressor in another due to different targets and mechanisms of action (Croce, 2009). Accordingly, this miRNA may be found upregulated in some cancer types, where it acts as oncogene, but downregulated in other cancers, indicative of tumor-suppressor function. An example is represented by miR-222/221 cluster that is overexpressed in breast, lung, or liver cancers where targets important tumor suppressors such as PTEN, p27, p57, while the same cluster is downregulated in erythroblastic leukemias where target c-KIT oncogene (Garofalo et al., 2012). The causes of the widespread misexpression of miRNAs in cancers can be explained by different mechanisms including: (a) chromosomal alterations of the miRNA genes, (b) DNA point mutations, (c) epigenetic mechanisms, (d) transcriptional modulation, or (e) genetic and epigenetic alterations in the transcriptional and post-transcriptional machinery responsible for miRNA production (Di Leva and Croce, 2010). Despite the large scientific interest for the understanding of miRNA dysregulation in cancer, the most daunting task is still the discovery of the biological functions of the dysregulated miRNAs in cancer. One main rule is emerged from the vast literature about the biological activity of miRNAs in cancer: oncogenic miRNAs repress the expression of tumor-suppressor genes, while tumor-suppressor miRNAs repress the expression of oncogenes (Esquela-Kerscher and Slack, 2006). For example, overexpression of the oncogene, miR-21, frequently highly expressed in solid and hematologic malignancies, represses strong tumor suppressors as PTEN or programed cell death 4 (PDCD4) while loss of the tumor-suppressor miR-15a/miR-16-1 in CLL induces the overexpression of the anti-apoptotic BCL2 (Cimmino et al., 2005; Meng et al., 2007; Asangani et al., 2008). Another common mechanism of miRNA activity in cancer cells is their involvement in negative and positive feedback loops. This is well illustrated by miR-146a, which is transactivated by the NF-κB pathway and negatively feeds back on this signaling cascade by targeting two upstream activators of the pathway, TRAF6 and IRAK1 (Taganov et al., 2006). Interestingly, deletion of miR-146a in mice results in increased activity of NF-κB in splenocytes and the consequent development of NF-κB-dependent myeloid sarcomas (Zhao et al., 2011). Finally, a particularly intriguing, but poorly understood, aspect of the biology of miRNAs is their presence in numerous body fluids, including serum, plasma, saliva, and amniotic fluid (Cortez et al., 2011). miRNAs in serum correlate with the presence of hematologic malignancies and solid tumors and have been reported to be of value for early detection of various types of cancer, preceding diagnosis by conventional methods (Boeri et al., 2011). The question of whether tumor-associated miRNAs detected in circulation results from tumor cell death and lyses, or instead from secretion by tumor cells remains unanswered. It has been reported that the profile of secreted miRNAs does not reflect the miRNA composition of the primary tumor, suggesting active regulation of miRNA release or cellular retention (Collino et al., 2010). Generally, miRNAs are present in biological fluids as lipoprotein complexes, small membranous vesicles known as exosomes or as non-vesicular Ago2 ribonucleoprotein complexes (Arroyo et al., 2011).

**Table 1:** **Common miRNAs altered in human cancers**.

MicroRNA	Expression in cancer	Function	Mechanism of deregulation	Targets
Let-7a-2	Down in breast, lung, colon, ovarian, and stomach cancer	Tumor suppressor	Repressed by MYC	KRAS, HMGA2, MYC, DICER, BCLXL, IMP-1, CDC34, IL6
miR-15/16	Down in CLL, prostate cancer, and pituitary adenomas	Tumor suppressor	Genomic loss, mutated, activated by p53	BCL2, COX2, CHECK1, CCNE1, CCND1, CCND2, BMI-1, FGF2, FGFR1, VEGF, VEGFR2, CDC25a
miR-29 family	Down in AML, CLL, lung and breast cancer, lymphoma, hepatocarcinoma, rhabdomyosarcoma	Tumor suppressor	Genomic loss, activated by p53, repressed by MYC	CDK6, MCL1, TCL1, DNMT1, DNMT3a, DNMT3b
miR-34 family	Down in colon, lung, breast, kidney, and bladder cancer	Tumor suppressor	Repressed by MYC	SIRT1, BCL2, NOTCH, HMGA2, MYC, MET, AXL. NANOG, SOX2, MYCN, SNAIL
miR-26a	Down in liver cancer	Tumor suppressor	Repressed by MYC	CCND2, CCNE2
miR-200 family	Down in aggressive breast and ovarian cancer	Tumor suppressor	Repressed by ZEB1/2	ZEB1, ZEB2, BMI-1, SUZ-12, FN1, LEPR, CTNNB1, JAG1, MALM2, MALM3, p38 alpha
miR-155	Up in high risk CLL, AML, breast, lung, colon cancer, and lymphoma	Oncogene	Activated by NF-KB	SOCS1, BACH1, MEIS1, ETS1, FOXO3A, hMSH2, hMSH6, hMLH1, SMAD5, WEE1, SHIP1, CEBPB
miR-21	Up in lung, breast, pancreas stomach, ovary prostate cancer, and CLL, AML, glioblastoma, myeloma	Oncogene	Activated by IL6, GF1alpha	PTEN, TPM1, PDCD4, SPRY1, TIMP3, RECK
miR-221/-222	Up in invasive ductal carcinoma, lung cancer, hepatocellular carcinoma, papillary thyroid cancer	Oncogene	Activated by MET in lung cancer; repressed by ERalpha in breast; activated by PLZF in melanoma; activated by NF-Kb and cJun in prostate cancer and glioblastoma cells	p27(Kip1), p57(Kip2), PTEN, TIMP3, FOXO3A, ERalpha, KIT, TRSP1, DICER, APAF1, PUMA, PTPμ
miR-17/92	Up in lung, breast, colon	Oncogene	Activated by E2F1 and MYC	PTEN, BIM, HIF1, PTPRO, p63, E2F2, E2F3, TSP-1, CTGF, p21(WAF1), JAK1, SMAD4, TGFbetaII, MnSOD, GPX2, TRXR2

## miRNA as Diagnostic Tools in Ovarian Cancer

Genome-wide miRNA profiling techniques have shown their utility to classify tumors based on their origin and differentiation state and to help in diagnosis and prognosis. As discussed above, several reports have already shown this miRNA feature for several tumor types. The first report of miRNA dysregulation in ovarian cancer came from our laboratory in 2007: miRs expression profiles were shown to discriminate between ovarian-cancer specimens and normal ovaries (Iorio et al., 2007) (Table 2). miR-200a and miR-141 were identified as highly upregulated in cancer, whereas miR-199a, miR-140, miR-145, and miR-125b1 were most significantly downregulated. In this study, specific miRNA deregulation was also used to differentiate the histological subtypes of ovarian carcinomas. For example, miR-200a and miR-200c were upregulated in all subtypes (mucinous, endometrioid, and clear cells), miR-200b and miR-141 were upregulated in serous as well as endometrioid carcinomas, and miR-21, miR-203, and miR-205 were upregulated only in endometrioid carcinomas. Indeed, miR-145 was downregulated in serous and clear-cell carcinomas, while miR-222 was downregulated in both endometrioid and clear-cell carcinomas. Later, Coukos laboratory highlighted a large down-regulation of miRNAs in ovarian-cancer cell lines and cancer specimens (Zhang et al., 2008). The authors identified a different expression of 44 miRNAs between early- and late-stage ovarian cancer with a complete down-regulation for all miRNAs in late-stage tumors. These signatures included three known tumor-suppressors miRNAs, mir-15a, mir-34a, and mir-34b. The authors also showed that the region containing the up-regulated miR-182 was amplified in 28.9% of ovarian carcinomas, whereas, miR-15a was deleted in 23.9% of ovarian carcinomas, as previously also shown for CLL (Calin et al., 2002). Further genome-wide miRNA studies were performed and all defined a large miRNA dysregulation in ovarian tumors. To date, Nam et al. (2008) identified 23 aberrantly expressed miRNAs in at least 60% of ovarian-cancer samples with miR-21 as the most upregulated (85% samples) and miR-125b (95% samples) most down-regulated miRNAs. Yang et al. (2008a) identified 36 miRNAs differentially expressed between normal ovarian cells and tumors, including miR-199a*, miR-214, miR-200a which were found upregulated in 53, 56, and 43% tumor tissues respectively, and associated with high-grade and late-stage tumors. miR-100 was identified instead as downregulated in 76% of tumors. In contrast with these data, Eitan et al. (2009) identified miR-200a, miR-34a, and miR-449b as the most down-regulated miRNAs in the advanced (stage III) ovarian tumors with miR-200a associated in the early-stage disease to an improved overall survival. miR-200a was also identified as predictor of favorable outcome in another profiling study of a cohort of 55 advanced ovarian tumors (Hu et al., 2009). Another member of the miR-200 family, miR-200c, was also identified by Marchini et al. (2011) as associated with progression-free survival, overall survival, or both in multivariate analysis of stage I ovarian cancers. In a later study in 2011, The Cancer Genome Atlas (TCGA) provided the first comprehensive molecular classification of a large cohort of high-grade serous ovarian carcinomas by integrated analyses of multidimensional data, including miRNA expression profiles, to identify molecular abnormalities that influence ovarian-cancer pathophysiology, affect outcome, and constitute therapeutic targets. Transcriptomic analyses identified four molecular subtypes of ovarian cancer, not significantly associated to survival, named Immunoreactive, Differentiated, Proliferative, and Mesenchymal based on the enrichment of specific genes in the subtype. miRNA expression instead differentiated the tumor specimens in three main subtypes where miRNA subtype 1 overlapped with the mRNA Proliferative subtype and miRNA subtype 2–3 overlapped with the mRNA Mesenchymal subtype. The subtype 1 was associated with worse patient survival as compared to the other two subtypes. A recent elaboration of the TCGA data has been performed by Dr. Zhang laboratory (Yang et al., 2013). The authors showed that integrated analysis of miRNAs and transcriptome is able to group the transcriptional subtypes into two more clinically relevant subtypes, one mesenchymal and one epithelial. The analyses highlights the important role of a miRNA regulatory network consisting of eight key miRNAs for the mesenchymal subtype including miR-141 and miR-200, miR-29c, miR-101, miR-506, and miR-128.

**Table 2:** **miRNA profiling studies in human epithelial ovarian cancers**.

Reference	Number of samples/subtypes	Method of analyses	Main findings
Iorio et al. (2007)	15 Normals/69 tumors 31 Serous/8 endometrioid/4 clear cells/9 poorly differentiated/1 mucinous	miRNA microarray	Ovarian cancer-specific miRNA signature Subtypes specific miRNA signature Epigenetic mechanism responsible for their aberrant expression
Yang et al. (2008a)	10 Tumors and 10 “normal” HIOSE cell line	miRNA microarray	Ovarian cancer-specific miRNA signature miR-214 induces cell survival and cisplatin resistance through targeting PTEN
Laios et al. (2008)	3 Primary serous/3 recurrent serous tumors	qRT-PCR	miR-9 and miR-223 can be biomarkers in recurrent ovarian cancer
Nam et al. (2008)	22 Serous tumors/8 normals	miRNA microarray	Ovarian cancer-specific miRNA signature
Zhang et al. (2008)	106 Tumors 109 Tumors 76 Tumors 504 Tumors	miRNA microarray, aCGH, affymetrix cDNA microarray, tissue array,	miRNAs are downregulated in malignant transformation and tumor progression Genomic copy number loss and epigenetic silencing account for miRNA dysregulation
	96 Tumors	qPCR validation
Dahiya et al. (2008)	34 Tumors and HOSE-B cell line	miRNA microarray	Ovarian cancer-specific miRNA signature
Sorrentino et al. (2008)	Drug-resistant vs. wild-type cancer cell lines	miRNA microarray	Paclitaxel and cisplatin resistance is associated with a specific miRNA fingerprint
Yang et al. (2008b)	69 Tumors (42 sensitive/27 resistant)	miRNA microarray	Let-7i is a modulator of platinum-based chemotherapy Let-7i is a biomarker to predict chemotherapy response and survival
Boren et al. (2009)	16 Ovarian cancer cell lines	miRNA microarray	miRNA signature associates to cell line drug response
Wyman et al. (2009)	33 Tumors/HOSE-B cell line	Deep sequencing	Ovarian cancer-specific miRNA signature
			Subtypes specific miRNA signature
Eitan et al. (2009)	19 Tumors (stage I)/38 tumors (stage III)	miRNA microarray	miRNA signature during progression miRNA expression associated with response to platinum-chemotherapy
Hu et al. (2009)	55 Advanced-stage tumors	miRNA microarray	miR-200b-429 are biomarkers for ovarian cancer outcome
Lee et al. (2009)	33 High-grade serous tumors 2 Low-grade serous tumors	miRNA microarray	No abnormalities in miRNA expression correlated to BRCA1/2 status
	2 Serous borderline tumors		miR-34c and miR-422b are prognostic biomarkers
	3 Normal fallopian tubes	
Nagaraja et al. (2010)	10 Human clear-cell ovarian cancer cell lines and 1 normal ovarian surface epithelial cultures	Deep sequencing	Clear-cell ovarian cancer-specific miRNA signature miR-101 inhibits mTOR pathway and increases rapamycin sensitivity
Creighton et al. (2010)	8 Serous tumors 4 Serous cancer cell lines 4 NOSE cell lines	Deep sequencing	miR-31 is downregulated in cancer Reduced levels of miR-31 are correlated with defects in the p53 pathway
Vaksman et al. (2011)	21 Tumors (13 effusions/8 primary tumors)	miRNA microarray	miRNA signatures for the primary tumors and effusions
Kim et al. (2010)	103 Tumors	miRNA microarray	miRNA signature is correlated with clinico-pathological parameters (subtype, grade, survival)
Marchini et al. (2011)	144 Tumors (stage I)	miRNA microarray	Ovarian cancer-specific miRNA signature
			miR-200c is a predictor of survival and relapse
Cancer Genome Atlas Research Network (2011)	489 Serous tumors	miRNA microarray	Global analyses of mRNA expression, miRNA expression, promoter methylation, and DNA copy number

MicroRNAs signatures have demonstrated their potential as diagnostic tool also in the ability to predict the clinical response to chemotherapy. In 2008, again in collaboration with our laboratory, Dr. Zhang’s group identified the involvement of let-7i in response to cisplatin for the treatment of ovarian cancer (Yang et al., 2008b). Another study performed by Eitan et al. (2009) analyzed the miRNA correlation to platinum-based chemotherapy response in stage III patients. By comparing the miRNA expression between patients that achieved complete response with no recurrence within 6 months of the end of treatment and patients that progressed really rapidly after treatment, the authors identified seven miRNAs to be significantly differentially expressed, including hsa-miR-27a, 23a, miR-378. The differential expression of these three miRNAs between sensitive and resistant tumors was also observed in the subset of stage III patients treated by the combined paclitaxel/carboplatin treatment. Leskelä et al. (2010) demonstrated instead that miR-200 family showed a significant association with treatment response to paclitaxel–carboplatin regimen: women lacking complete response to paclitaxel–carboplatin regimen had tumors with significantly lower miR-200c levels than the ones who had achieved complete response; in addition, higher expression of miR-200c was associated with lower relapse/progression rates. Currently, a combined treatment of carboplatin/paclitaxel has been adapted as the standard treatment for women with advanced epithelial ovarian cancer (EOC) (Hiro et al., 2010). However, many patients with ovarian cancer which initially respond to chemotherapy eventually relapse with drug-resistant disease (Hassan et al., 2011). Acquired chemoresistance is a major obstacle for successful cancer treatment. Based on the correlation between drug response and miRNA expression, many studies have tried to manipulate the mechanisms responsible for chemoresistance by altering the levels of miRNAs. For example, Liu et al. (2012) have demonstrated that a chimera composed of a MUC1 aptamer and let-7i can efficiently deliver let-7i into paclitaxel/cisplatin resistant ovarian tumor cells and subsequently resensitize to the apoptotic role of the drugs the ovarian malignant cells. Prislei et al. (2013) showed that overexpression of miR-200c repressed the expression of level of class III β-tubulin (TUBB3), a factor associated with drug resistance and poor prognosis in ovarian cancer, and increased sensitivity to paclitaxel and cisplatin. Same results were also obtained by Cochrane et al. (2010) which showed that restoration of miR-200c increases sensitivity to microtubule-targeting agents and mitigates invasiveness by 85%. Two other studies reported that miR-182 and miR-125b conferred resistance to cisplatin, possibly by their anti-apoptotic activity due to the repression of two important tumor suppressors, PDCD4 and Bcl-2 antagonist killer 1 (Bak1), respectively (Kong et al., 2011; Wang et al., 2013).

Because the majority of ovarian-cancer patients are diagnosed with advanced-stage disease, identification of early tumor is essential to improve prognosis and therapy. One of the best ways to early diagnose, aid prognosis, and predict therapeutic response is by using diagnostic or prognostic serum and tissue biomarkers. Unfortunately, there are not many reliable serum biomarkers for ovarian-cancer currently used in the clinic, and tissue-based markers require an invasive procedure to obtain samples. Therefore, new efforts are needed to identify new serum markers to aid in the screening process. The ability to profile miRNAs in circulation have shown a non-invasive opportunity to identify promising alternative approaches to the current strategies for ovarian-cancer surveillance and early diagnosis. In this context, by using serum samples from patients with various stages of ovarian cancer, Taylor and Gercel-Taylor (2008) showed that 46% of miRNAs in the exosomes were the same as those in the primary tumors. Twelve miRNAs were present at a higher proportion in malignant cells (es: mir-155, -29), while 31 were present at elevated levels exclusively in exosomes (es: miR-203, -205). A study from our laboratory identified 23 miRNAs differentially expressed in serum of patients with ovarian cancer; only 10 of these miRNAs were in common with miRNAs that have been previously published in the literature as part of the miRNA signatures of ovarian cancer (including mir-21) (Resnick et al., 2009). In another study, the levels of four miRNAs (miR-200a, b, c, and miR-182) were identified as differentially expressed between the serum of 28 patients with serous ovarian cancer and healthy age-matched volunteers (Kan et al., 2012). miR-200c was the most differentially expressed and a combination of miR-200b and miR-200c gave the best predictive power for serous ovarian cancer. A different approach was instead taken by Vaksman et al. (2011) who analyzed the miRNA expression profiles of primary ovarian cancers and effusions from patients with disease spread beyond the ovary in order to define a new parameter for metastatic dissemination. The authors identified three groups of miRNAs: (1) highly expressed in primary ovarian cancer and effusions; (2) overexpressed only in primary ovarian cancer; and (3) overexpressed only in effusions. miR-210, -182, and -99a were significantly overexpressed in effusions compared to primary tumors, whereas hsa-miR-145 was significantly overexpressed in primary carcinomas. Overall, the above studies provided useful biomarkers information for ovarian cancer. The large heterogeneity of the results, based on differences in the samples analyzed and technology applied, highlights that additional studies are needed to define predictive and reliable miRNA signatures that can find a clinico-pathological application.

## Cause of miRNA Dysregulation in Ovarian Cancer

An important aspect of miRNA biology in ovarian cancer that has been taken in consideration during the last few years is the cause of the large dysregulation of miRNAs in cancer that profiling studies have shown. First, chromosomic alterations have been identified for several miRNA genes. As previously described, Coukos’s laboratory identified a consistent amplification of miR-182 region and deletion of miR-15 in ovarian carcinomas (Zhang et al., 2008). The same authors also showed a remarkably high frequency of miR-210 gene copy deletions in ovarian-cancer patients, and that gene copy number correlated with miR-210 expression levels (Giannakakis et al., 2008). Loss of heterozygosity at the let-7a-3/let-7b and mir-143/mir-145 loci was also detected in 50 and 22% of 90 ovarian carcinomas, respectively (Bearfoot et al., 2008). The authors analyzed also the somatic mutations status of a ∼500-bp genomic region surrounding 10 ovarian-cancer-implicated miRNA genes (let-7a-2, let-7a-3, let-7b, miR-10b, miR-125b-1, miR-125b-2, miR-143, miR-145, miR-200c, miR-206). Despite analyzing a large cohort of primary tumors, no somatic mutations were detected at the genomic regions corresponding to the primary, precursor, or mature miRNAs in any of the miRNA genes studied, suggesting that somatic mutations may not be a common mechanism of miRNA inactivation in ovarian cancer. Another mechanism that has been analyzed to explain the miRNA dysregulation in ovarian cancer is the altered levels or presence of mutations in the main enzymes of the miRNA biogenesis machinery, such as Dicer and Drosha. In fact, aberrations of the main proteins that are involved in miRNA processing will lead to changes in miRNA expression and ultimately to alterations of miRNA-mediated gene regulation. A work published in 2010 evaluated a decrease of 60 and 51% in the levels of Dicer and Drosha mRNAs, respectively, in 39% of ovarian-cancer tissues analyzed (Merritt et al., 2008). The authors also showed that, neither Dicer nor Drosha mRNA levels were significantly associated with age, tumor grade, or response to chemotherapy but low Dicer and Drosha mRNA levels were, however, significantly associated with advanced tumor stage or suboptimal cytoreductive surgery, respectively. Moreover, women whose tumor had low levels of Dicer and Drosha mRNA showed a reduced overall survival, indicating a clinical relevance for an alteration in the levels of Dicer and Drosha mRNAs in ovarian-cancer cells. Same conclusion were also obtained by another study performed by Pampalakis et al. (2010) who observed a marked down-regulation of Dicer expression in ovarian tumors of higher grade and higher stage. Unfortunately, the basis of the observed down-regulation of Dicer or Drosha expression in ovarian tumors is unknown. We may speculate that the presence of a large CpG island at Dicer genomic loci indicates that genomic DNA methylation may account for Dicer down-regulation in ovarian tumors, but further investigations are needed.

An intriguing report came from Dr. Huntsman laboratory which discovered the presence of recurrent somatic missense mutations of DICER1 in non-epithelial ovarian tumors (Heravi-Moussavi et al., 2012). These mutations were predominantly restricted to a specific subset of non-epithelial ovarian tumors and highly prevalent (60%) in Sertoli–Leydig cell tumors. The recurrent and focal nature of these mutations and their restriction to non-epithelial ovarian tumors suggested a common oncogenic mechanism associated with a specific altered DICER1 function that is selected during tumor development in these cell types. The localized and focal pattern of mutations is typical of dominantly acting oncogenes, like KRAS and BRAF. The absence of loss of heterozygosity that is seen in association with germline DICER1 mutations provides further evidence against a role for DICER1 as either a haploinsufficient or a two-hit recessive tumor suppressor in this non-EOC. We can imagine that the new mutated DICER1 alleles produce viable protein that is able to create a different miRNA profile with oncogenic potentials. As well as for Dicer and Drosha, Vaksman, and collaborators suggested a role in tumor progression of ovarian cancer for the Ago family members, Ago1 and Ago2. Specifically, the authors identified an overexpression of Ago1 and Ago2 in the peritoneal effusions compared with primary ovarian carcinomas, and high levels of Ago2 mRNA in solid metastases compared with primary tumors Vaksman et al., 2012).

Based on high-throughput results, Zhang et al. (2008) showed that if deletions occur in up to 15% of genomic loci harboring miRNAs that are downregulated, at least one-third of down-regulated miRNAs may be silenced by epigenetic alterations. Iorio et al. (2007) showed that 11 miRNAs, including miR-21, miR-203, miR-146b, miR-205, miR-30-5p, and miR-30c as the most significantly induced, are differentially expressed after treatment with the demethylating agent 5-AZA. Lu et al. (2007) showed that let-7a-3 is methylated in EOC, and low expression of let-7a is associated with poor prognosis. Epigenetic silencing of miR-130b through hypermethylation of the adjacent CpG island has been also identified and low expression of miR-130b was correlated to ovarian cancer with high stage and multidrug resistance (Yang et al., 2012). In fact, treatment of ovarian-cancer cells with demethylating agents increased miR-130b levels and decreased the IC50 of paclitaxel and cisplatin treatment. Complementary mechanisms, including transcriptional regulation, may also cooperate in miRNA deregulation of ovarian cancer. An important example of miRNA transcriptional control in ovarian cancer is represented by the miR-200 family, which has been shown highly modulated in ovarian cancer. The miR-200 family contains miR-200a, miR-200b, miR-200c, miR-141, and miR-429 which are arranged in two clusters in the human genome. miR-200a, miR-200b, and miR-429 are located on chromosome 1, while miR-200c and miR-141 are on chromosome 12. ZEB1/2, two transcription factors involved in the mediation of the epithelial to mesenchymal transition, can inhibit the expression of miR-200 family members by binding to the promoter of both miR-200 clusters thereby blocking transcription (Gregory et al., 2008). In turn, over expression of miR-200 family members repress ZEB1/2 levels, and leads to higher levels of E-cadherin and an epithelial phenotype (Burk et al., 2008). In fact, Park et al. (2008) have shown a positive correlation in the expression of E-cadherin with the expression of miR-200c in ovarian-cancer tissues. We can summarize that cancer cells after being triggered by molecular signaling, such as TGF-β or PDGF-D, increases their levels of ZEB1/2 which in turn decrease the expression of miR-200 and induce EMT. An interesting example of multi mechanism control of miRNA expression in ovarian cancer is represented by the miR-34 family. miR-34 clusters are part of the transcriptional program activated by p53 (He et al., 2007). Mutational and loss of TP53 function is one of the most frequent genetic abnormalities in ovarian cancer and is observed in 60–80% of both sporadic and familial cases (Bast et al., 2009). In accordance with the loss of TP53, miR-34 members (miR-34a, b, c) have been found strongly repressed in ovarian cancer: miR-34a expression is decreased in 100% and miR-34b*/c in 72% of EOC with p53 mutation (Corney et al., 2010). However, miR-34a was also downregulated in 93% of tumors with wild-type p53, indicating the presence of other mechanisms implicated in the suppression of miR-34a gene. In fact, the authors identified methylation and reduced copy number at the mir-34a gene in 27 and 39% of ovarian-cancer tissues, respectively.

## Conclusion

In the next 5 years we could witness a very exciting periods for drug development in ovarian cancer since the introduction of cisplatin into chemotherapy. The discovery of aberrantly expressed miRNAs in ovarian cancer have defined new pathways in ovarian tumorigenesis and progression. miRNA expression profiles in tissues and biological fluids can potentially be used for the detection and surveillance of ovarian cancer. But miRNAs have also shown their efficacy in altering the sensitivity to traditional drugs. Therefore, targeted therapies should be accelerated by the delivery of specific miRNAs or miRNA inhibitors, which have been shown to be effective in ovarian-cancer cells.

## Conflict of Interest Statement

The authors declare that the research was conducted in the absence of any commercial or financial relationships that could be construed as a potential conflict of interest.
